The article "Investigating the Impact of Transportation Infrastructure and Tourism on Carbon Dioxide Emissions in China" was retracted in 2023. Reasons: unreliable results or conclusions; concerns about the data; concerns about the peer review; concerns about the citations.

# Investigating the Impact of Transportation Infrastructure and Tourism on Carbon Dioxide Emissions in China

**DOI:** 10.1155/2022/8421756

**Published:** 2022-09-09

**Authors:** Qiang Zhang

**Affiliations:** Economic Management School, Baoji University of Arts and Sciences, Baoji, Shaanxi 721013, China

## Abstract

In order to effectively address or eliminate the impact of CO_2_ emissions, it is essential to investigate the analysis of CO_2_ emissions under transport infrastructure and tourism. Transportation infrastructure helps to achieve carbon dioxide emission limitation, which is crucial for resource distribution, effectively summarizing the regularity and innovation in the process of carbon dioxide emission limitation. In the case of fully grasping the principles of low-carbon tourism development and related policy protection, a suitable low-carbon tourism development model is found. By constructing a data analysis model, this paper analyzes the impact of transportation infrastructure and ecotourism on carbon dioxide emission limitation. In terms of methods and systems, effective measures are given to the role of Chinese traffic settings in tourism, and the carbon emission system of the entire life cycle of traffic settings is analyzed, and the boundary of the impact of traffic carbon emissions on tourism is determined. In response to this problem, it is necessary to reform and optimize the transportation facility of the carbon emission accounting method, which has a positive effect on the green development and low-carbon development of the Chinese economy for ecotourism and transportation infrastructure.

## 1. Introduction

With the continuous development of social economy, tourism is also booming. With the improvement of people's living standards and the continuous changes in social awareness and ideas, travel has become the norm in daily life. Even in the past few years, there has been a boom in overseas travel, and tourism has become a rigid demand. But what follows is the emergence of new problems, such as littering in scenic spots, destruction of historical sites and facilities in scenic spots, and other nonenvironmental and uncivilized behaviors. Therefore, it is an urgent problem and focus to analyze the influencing factors of tourists' environmental protection behavior and to continuously instill and integrate the concept of environmental protection into the conscious behavior of citizens. The behavior of environmental protection is also called environmental low-carbon behavior and environmental protection behavior in China [1–3]. At present, the research of environmental protection awareness by experts within the industry mainly focuses on the influence of demographic factors such as the age, education level, and birth environment of citizens, as well as subjective environmental ecological education, environmental attitude, and environmental protection awareness or from the perspective of tourism motivation. Current environmental behavior interventions mainly focus on propaganda, punishment, and other programs but have not paid attention to the impact of traditional Chinese culture and reward and punishment measures on environmental behavior [4–6]. Carbon dioxide emission reduction behavioral influencer analysis and real-time risk alerts are also effective data collection and analysis processes for transport infrastructure and tourism. Collect indicator data from the ecological environment and give feedback to monitoring personnel. Ecological environment detection and real-time risk monitoring are of great significance for ecological environment-related resource distribution, flow planning service level, and safety monitoring. The analysis of factors affecting carbon dioxide emission reduction behavior and real-time risk alerts are important manifestations of ecological environment management and systematic integration, providing detailed data information for the operation and maintenance of the ecological environment. In terms of capacity planning, eco-environmental performance analysis, abnormal monitoring, link status monitoring, and capacity planning play an important role. As the focus of current research in this field, the analysis of influencing factors of carbon dioxide emission reduction behavior can be perfectly combined with different industries, and the data of different industries can be fully used in the actual analysis environment of carbon dioxide emission reduction behavior influencing factors. With the growth of tourism, people's requirements for carbon emissions are also more demanding, but most researchers still stay at the linear level of research, and only a few researchers have carried out the deepening of the nonlinear level [7–9]. There is no research on the nonlinear level of the tourism development level and tourism development speed, and these two are the decisive reasons. Carbon emission reduction of transportation infrastructure involves many fields such as raw material production, raw material transportation, and building construction and involves related engineering construction and environmental protection management departments. There are certain overlapping and blank responsibilities, management is difficult, and the effect of carbon emission management is not ideal. In the implementation stage, the emission reduction needs to be maximized. The Chinese environment studies have entered a new course. The differences in the economic development and economic situation of each place have a decisive factor on the local carbon emissions. Change and role require lower carbon, greener, and less energy loss to generate maximum tourism. Due to the large differences in regional economic growth, according to the regional economic development level and carbon dioxide emissions of each country, based on the actual situation, the reasonable and scientific carbon emission reduction policy standards are formulated, which has become the first choice for the development of low-carbon economy in China. When formulating low-carbon emission reduction policies, countries need to effectively consider their own economic development, resource availability, and green relevant policies aiming at different regions, areas, and corresponding urban resources, actively encourage the country to actively explore the allocation of carbon dioxide emissions and renewable resources suitable for its own region, and guide the whole society to save resources, improve resource efficiency, and reduce environmental pollution. The key to the sustainable growth of the proposed tourism development is to break through the tourism structure. Through the analysis from the perspective of resources, it is actually the current regulations of the current environment to find the form of green tourism and green environment. Facts have proved that the development of tourism in this country is inseparable from the country's carbon emissions and the environment, especially for the huge country [10, 11]. Through two levels of analysis, the first level is that the tourism resources of each country in our country are disparate, the development of each country and each region also has a large gap, and the country needs to manage carbon emissions while taking into account the growth of tourism. The second level is that each country has its own development characteristics, such as the development track of industry, tourism, and cities; therefore, the issue of carbon emissions is not summarized at one level, but there is a special relationship between the development of tourism and emission reduction, and this consequence can also be seen in each country's own characteristics. Considering the implementation of carbon emissions according to one standard leads to a different picture of results. So, how to maintain the normal growth of tourism while ensuring the emission of carbon emissions? This is a problem that every country needs to solve so that both can develop in a balanced way. Therefore, it is necessary to analyze the different levels of each region and the tourism situation. According to the analysis results, we will find a solution to fundamentally solve the contradiction between tourism and carbon emissions between countries. The solution of this problem will also bring more long-term benefits to the country [12, 13].

The article "Investigating the Impact of Transportation Infrastructure and Tourism on Carbon Dioxide Emissions in China" was retracted in 2023. Reasons: unreliable results or conclusions; concerns about the data; concerns about the peer review; concerns about the citations.

The global temperature has gradually warmed up, which is related to the emission of carbon dioxide. Total carbon dioxide emissions have increased by 30 percent over the past decade, 25 percent of which comes from urban transport carbon emissions. The resource consumption of transportation is also quite large, and these data have already caused a great threat to the urban environment, and there is an adverse impact in the era of the development of the human and self-heating industry. Through this worrying environment, the world is creating new opportunities for resource development. The term low-carbon transportation also appears in people's ideas, and of course it is the goal that every city in the world needs to achieve. This paper analyzes the carbon emission situation of Chinese transportation installations through research on the existing transportation carbon emission calculation in China and foreign countries, and at the same time, corresponding measures are put forward based on the existing traffic settings, which provides strong support for the development of healthy and low-carbon transportation in China.

## 2. Basic Knowledge and Related Calculation Methods

Ecotourism plays a very important role in the promotion of green economy in China. Ecotourism promotes transportation infrastructure and effectively reduces the consumption of carbon dioxide per unit. The development of the economy has made the transportation infrastructure continue to intensify, resulting in an increase in carbon dioxide emissions, and the increase in consumer demand has increased carbon dioxide emissions. The realization of real-time, rational, and precise monitoring of carbon dioxide emissions can also provide a theoretical basis for the decision analysis of relevant environmental protection inspection departments, which is of great significance to the emergence of more transportation infrastructure projects. A detailed analysis of the transportation infrastructure is carried out to explore the problems and shortcomings of the carbon dioxide emission process so that the training and improvement plan can be formulated later. There are many differences in carbon dioxide emissions among countries and the corresponding reasons. There are many differences in CO_2_ emissions between countries, and the basis of this classification is not only based on the boundaries of tourism areas, nor is the high or low standard set by the size of CO_2_ emissions, but the classification should take into account the tourism situation, the rate of tourism development and growth patterns [14, 15]. The situation, the speed of tourism development, and the way of growth should be comprehensively considered. It can be concluded that due to the large differences in the development of tourism in different countries, according to the level of tourism development and carbon dioxide emissions in each country and according to the actual situation, reasonable and scientific carbon emission reduction policy standards are formulated, which has become the preferred way for countries to develop low-carbon tourism. When formulating low-carbon emission reduction policies, the premise is to consider the basic situation of tourism development in different countries, the basic resources of different regions and corresponding cities, the current situation of environmental pollution and characteristics of industrial structure, as well as relevant legal policies, and actively encourage countries to boldly explore their own ways of allocating carbon dioxide emissions and renewable resources to guide the whole society to save resources, improve resource efficiency, and reduce environmental pollution. As shown in Figure 1:

As an emerging tourism body in China with a relatively high degree of openness in tourism development, the emergence of Chinese trade and investment protectionism will lead to the slow development of its tourism trade and will seriously affect financial financing. The continuous development of various factors such as big data, artificial intelligence, and blockchain will make more traditional industries change continuously [15, 16]. At present, with the development of financial technology, different types of electronic payment models have begun to develop on a large scale. Using the characteristics and typical activities of LCA structure and transportation infrastructure construction, the carbon emissions generated in the process of transportation infrastructure are more vulnerable to extreme weather and sea level rise than developed countries (regions). After extreme weather events, the repair or reconstruction of damaged infrastructure not only hinders disaster relief work and economic recovery but also further consumes limited financial resources. The carbon dioxide emission management control strategy model and decision-making process are shown in Figure 2.

The article "Investigating the Impact of Transportation Infrastructure and Tourism on Carbon Dioxide Emissions in China" was retracted in 2023. Reasons: unreliable results or conclusions; concerns about the data; concerns about the peer review; concerns about the citations.

In the process of accepting the awareness of carbon dioxide emission reduction and environmental protection, tourists have experienced the process of learning, understanding, and accepting. The surrounding environment makes certain technical changes and adjustments to the subjective consciousness of tourists. When the probability of the corresponding environmental protection investment is adjusted, according to these random numbers, the judgment of tourists' awareness of carbon dioxide emission reduction and environmental protection is carried out, as shown in formula (1):

(1) $$\begin{array}{c} \text{tech ln vest}=\left\{\begin{array}{c} \text{tech ln vest}\left(t-1\right)-\Delta I_{1}\left(0\leq r<p^{d}\right),\\ \text{tech ln vest}\left(t-1\right)+\Delta I_{2}\left(p^{d}\leq r<p^{i}+p^{r}\right),\\ \text{tech ln vest}\left(t-1\right)\left(p^{i}+p^{r}\right)\leq r<1. \end{array}\right) \end{array}$$

Risk analysis results include the likelihood of transport infrastructure being exposed to specific catastrophic events and the consequences of such events. (2) shows the function that defines the risk that is widely used today.

(2) $$\begin{array}{c} R=\left\{S_{i},P_{i},D_{i}\right\},i=1,2,\ldots ,k, \end{array}$$

where *R* is the risk set; *S*_*i*_ is the damage factor set; *P*_*i*_ is the correlation probability of *S*_*i*_; *D*_*i*_ is the associated damage; *k* is the number of damage factors.

First of all, it is necessary to judge the ability of tourists. By constructing a corresponding model, using subjective constraints, discussing the relationship between input and output, and expressing it with a quantitative function, as shown in formula (3):

(3) $$\begin{array}{c} Q\left(t\right)=T\left(t\right)L^{\alpha }K^{\beta }. \end{array}$$

In the formula, *Q*(*t*) is the actual output quantity invested by tourists in period *t*, *T*(*t*) represents the technical level of tourists, awareness of carbon dioxide emission reduction, and environmental protection, and *L* is the labor input by corresponding environmental protection enterprises and training institutions, aiming to cultivate awareness of carbon dioxide emission reduction and environmental protection, *K* is the investment capital theory of environmental protection enterprises, and *α* and *β* are constants, as shown in the following formula:

(4) $$\begin{array}{c} T\left(t\right)=\frac{B-\text{tech ln vest}\left(t\right)}{1+B-\text{tech ln vest}\left(t\right)}. \end{array}$$

In order to further simplify the model, formula (5) is used to simulate the input cost of environmental protection enterprises, where *C*_1_ and *C*_2_ are constants:

(5) $$\begin{array}{c} \text{product Cost}=C_{1}\cdot Q\left(t\right)+C_{2}\cdot L. \end{array}$$

The operations of the *k*(*k*=1,2,…, *K*) group in the carbon dioxide emission analysis can be expressed as

(6) $$\begin{array}{c} s_{1}\left(t\right)=\sum_{m=0}^{M-1}\text{rect}\left(\frac{t-mT_{R}-kMT_{R}}{T_{p}}\right)\cdot \exp\left(j\pi \gamma {\left(t-mT_{R}-kMT_{R}\right)}^{2}\right)\\ \cdot \exp\left(j2\pi f_{sm}\left(t-mT_{R}-kMT_{R}\right)\right). \end{array}$$

In the formula, $t=\hat{t}+mT_{R}+kMT_{R}\left(m=1,2,\ldots ,M\right)$ represents the entire computing time, $\hat{t}$ represents the fast time, and tect(*u*) represents the corresponding rectangular window.

The article "Investigating the Impact of Transportation Infrastructure and Tourism on Carbon Dioxide Emissions in China" was retracted in 2023. Reasons: unreliable results or conclusions; concerns about the data; concerns about the peer review; concerns about the citations.

If the carbon dioxide emission analysis contains multiple feature points, then the coefficient of the backward feature of the *p*(*p*=1,2,…, *P*)th feature point can be expressed by *σ*_*p*_. If the corresponding time delay *τ*_*p*_(*t*) value of the characteristic point *p* in the transformation assistance in the carbon dioxide emission analysis does not change, then *τ*_*p*_(*t*) ≈ *τ*_*p*_(*t*_*m*,*k*_), *t*_*m*,*k*_=*mT*_*R*_+*kNT*_*R*_. At the same time, for the characteristic points of the carbon dioxide emission analysis, the *m*th subtransition assistance under the *k*th group of transportation infrastructure-assisted high-performance computing can be expressed as

(7) $$\begin{array}{c} s_{2}\left(\hat{t},m,k\right)=\sigma_{p}\text{rect}\left(\frac{\hat{t}-\tau_{p}\left(t_{m,k}\right)}{T_{P}}\right)\cdot \exp\left(j\pi \gamma {\left(\hat{t}-\tau_{p}\left(t_{m,k}\right)\right)}^{2}\right)\\ \cdot \exp\left(j2\pi f_{sm}\left(\hat{t}-\tau_{p}\left(t_{m,k}\right)\right)\right)+\varepsilon \left(\hat{t}\right). \end{array}$$

In the formula, *τ*_*p*_(*t*_*m*,*k*_)=2*R*_*P*_(*t*_*m*,*k*_)/*c*, *R*_*P*_(*t*_*m*,*k*_) are expressed as the instantaneous slope distance between the *p*th feature point and the emission limit analysis of carbon dioxide emission analysis, *c* is the speed of light, and $\varepsilon \left(\hat{t}\right)$ is represented as an additive constraint.

The definition of living welfare is based on the effective combination of consumption and the effective limitation of carbon dioxide emissions, the negative impact of emissions on the arrival of tourists' happy life, assuming that the expression of tourists' living welfare is

(8) $$\begin{array}{c} \max\int_{0}^{+\infty }\left(\ln\;C-\beta \;\ln\;P\right)e^{-\rho t}dt\text{.} \end{array}$$

In the expression, C represents the consumption of tourists, and *P* represents the stock of carbon dioxide. If *β* > 0 occurs, it represents the index of the impact of carbon dioxide emissions on tourists' lives, and if *ρ* > 0 occurs, it represents the index of tourists' patience. The carbon emission factors of commonly used resources and building materials are shown in Tables 1 and 2.

Substituting the total carbon dioxide emission function of expression (8) into expression (9), the average carbon dioxide emission can be obtained as follows:

(9) $$\begin{array}{c} \frac{\dot{P}}{Y}=\Omega {\left[\frac{Y}{A}\right]}^{\varphi }=\Omega L_{Y}^{\alpha \varphi }{\left[\frac{K}{A}\right]}^{\left(1-\alpha \right)\varphi }. \end{array}$$

The expression that can use the economic growth rate as the limiting condition of carbon dioxide emissions is

(10) $$\begin{array}{c} \frac{\dot{P}}{Y}=\delta^{-\varphi }{\left(1-\alpha \right)}^{\left(2\left(1-\alpha \right)\varphi \right)/\alpha }\Omega {\left(\delta L-\Omega \right)}^{\varphi }{\left(\rho +\Omega \right)}^{-\left(\left(1-\alpha \right)/\alpha \right)\varphi }. \end{array}$$

Substituting expression (9) into expression (8), the condition of carbon dioxide emission limit is expressed as a function. According to expression (9), the degree of influence of tourism on the economic growth rate can be realized. According to expression (10), it can be deduced that the CO_2_ emission limit varies with the economic growth rate. Therefore, according to the qualitative analysis, the use of tourism can realize the assessment of the impact degree of carbon dioxide emission limitation.

The article "Investigating the Impact of Transportation Infrastructure and Tourism on Carbon Dioxide Emissions in China" was retracted in 2023. Reasons: unreliable results or conclusions; concerns about the data; concerns about the peer review; concerns about the citations.

Through in-depth investigation and research of the formation of different carbon emission ranges, we can find measures and ways to reduce emissions. This effective measure is beneficial to the development of tourism in various countries. According to the difference between the current national carbon emissions and the development of tourism, this paper estimates and detects the transportation infrastructure through the proposed situation of “the role of tourism development on carbon emissions.” There is a single threshold between the level of tourism development and carbon emissions, and the level of tourism development directly affects the threshold in carbon emissions. There are obvious gaps in the relationship between tourism development and carbon dioxide emissions in different countries. Some data show that after calculating the total carbon emissions, each region is manually distinguished and studied through factors in different regions. Questions were raised about the arrangement of such predistinguished regions, which should be based on regional carbon emissions. Because of the interference of tourism, regular distinctions are made, and then distinctions are made according to the results and categories so that the carbon emission factors can be divided by region, and the relationship between tourism development and carbon emission growth changes can be studied, and it is recommended to effectively formulate and implement strategy of carbon reduction [17, 18].

## 3. Analysis of the Impact of Transportation Infrastructure and Tourism on Carbon Emissions

According to the sorting out of the key points of the carbon emission calculation of transportation infrastructure at home and abroad, there is currently no complete carbon emission quantitative calculation method system in the field of transportation infrastructure in China. There are inconsistent calculation boundaries, unclear calculation granularity, disordered methods, and lack of systematic management. There is a big gap with the carbon peak carbon neutralization target requirements [19, 20]. To develop Chinese overall tourism benefits and the concept of sustainable development, the first thing to solve is the situation of energy loss and carbon emissions. The nonlinear impact analysis structure of transportation infrastructure and ecotourism on carbon dioxide emissions is a finite-parameter linear model. On the basis of satisfying the finite parameter linear model, the finite parameter linear model can be used for optimization according to the steady-state ecological environment of the system. In the process of dynamic monitoring of the ecological environment, the nonlinear impact of transportation infrastructure and ecotourism on carbon dioxide emissions can be analyzed. According to the problems analyzed above, this paper uses the ecotourism demand function to express as follows:

(11) $$\begin{array}{c} w=\alpha L_{Y}^{\alpha -1}\int_{0}^{A}x{\left(i\right)}^{1-\alpha }\text{di}, \end{array}$$

(12) $$\begin{array}{c} p\left(i\right)=\left(1-\alpha \right)L_{Y}^{\alpha }x{\left(i\right)}^{-\alpha }. \end{array}$$

The obtained data are used for the analysis of the performance of the ecological environment protection, the operation status of the ecological environment protection, and the diagnosis of the cause of the failure and can also be used for the monitoring of the cause of the failure [11, 21].

The article "Investigating the Impact of Transportation Infrastructure and Tourism on Carbon Dioxide Emissions in China" was retracted in 2023. Reasons: unreliable results or conclusions; concerns about the data; concerns about the peer review; concerns about the citations.

Suppose the operation of group *k*(*k*=1,2,…, *K*) in the CO_2_ emission limit analysis can be expressed as follows:

(13) $$\begin{array}{c} s_{1}\left(t\right)=\sum_{m=0}^{M-1}\text{rect}\left(\frac{t-mT_{R}-kMT_{R}}{T_{p}}\right)\cdot \;\exp\left(j\pi \gamma {\left(t-mT_{R}-kMT_{R}\right)}^{2}\right)\\ \cdot \;\exp\left(j2\pi f_{sm}\left(t-mT_{R}-kMT_{R}\right)\right). \end{array}$$

In the formula, $t=\hat{t}+mT_{R}+kMT_{R}\left(m=1,2,\ldots ,M\right)$ represents the entire computing time, $\hat{t}$ represents the fast time, and tect(*u*) represents the corresponding rectangular window.

Assuming that carbon dioxide emission reduction is divided into *K* groups for sparse analysis, then the ecological transformation of consumption patterns in the *k*(*k*=1,2,…, *K*) group helps high-performance computing, which can be expressed as follows:

(14) $$\begin{array}{c} s_{1}\left(t\right)=\sum_{m=0}^{M-1}\text{rect}\left(\frac{t-mT_{R}-kMT_{R}}{T_{p}}\right)\cdot \;\exp\left(j\pi \gamma {\left(t-mT_{R}-kMT_{R}\right)}^{2}\right)\\ \cdot \;\exp\left(j2\pi f_{sm}\left(t-mT_{R}-kMT_{R}\right)\right). \end{array}$$

In the formula, $t=\hat{t}+mT_{R}+kMT_{R}\left(m=1,2,\ldots ,M\right)$ represents the entire computing time, $\hat{t}$ represents the fast time, and tect(*u*) represents the corresponding rectangular window.

If there are multiple feature points in the carbon dioxide emission reduction analysis, then the coefficient of the backward feature of the *p*(*p*=1,2,…, *P*) feature point can be expressed by *σ*_*p*_. If the corresponding delay value *τ*_*p*_(*t*) of the characteristic point *p* in the transformation boost of carbon dioxide emission reduction analysis does not change, then *τ*_*p*_(*t*) ≈ *τ*_*p*_(*t*_*m*,*k*_), *t*_*m*,*k*_=*mT*_*R*_+*kNT*_*R*_. At the same time, for the characteristic points of the carbon dioxide emission reduction analysis, the *m*th subtransformation assistance under the ecological transformation assistance of the *k*th group of consumption patterns under the high-performance computing can be expressed as follows:

(15) $$\begin{array}{c} s_{2}\left(\hat{t},m,k\right)=\sigma_{p}\text{rect}\left(\frac{\hat{t}-\tau_{p}\left(t_{m,k}\right)}{T_{P}}\right)\cdot \;\exp\left(j\pi \gamma {\left(\hat{t}-\tau_{p}\left(t_{m,k}\right)\right)}^{2}\right)\\ \cdot \;\exp\left(j2\pi f_{sm}\left(\hat{t}-\tau_{p}\left(t_{m,k}\right)\right)\right)+\varepsilon \left(\hat{t}\right). \end{array}$$

In the formula, *τ*_*p*_(*t*_*m*,*k*_)=2*R*_*P*_(*t*_*m*,*k*_)/*c*, *R*_*P*_(*t*_*m*,*k*_) is expressed as the instantaneous slope distance between the *p*th characteristic point and the emission evolution analysis of carbon dioxide emission reduction analysis, *c* is the speed of light, and $\varepsilon \left(\hat{t}\right)$ is the additive evolution. Then, for the transformation-assisted frequency modulation processing, we can set $\hat{f}=\gamma \left(\hat{t}-2R\left(t_{m,k}\right)/c\right)$, and then the carbon dioxide emission reduction analysis process is as follows:

(16) $$\begin{array}{c} s_{3}\left(\hat{f},m,k\right)=\sigma_{p}\text{rect}\left(\frac{\hat{f}}{\Delta f}\right)\exp\left(j\frac{4\pi }{c}\left(f_{sm}+\hat{f}\right)\Delta R\right)\cdot \exp\left(j\frac{4\pi }{c}\left(\Phi_{P}+\Phi_{B}\right)\right)+\varepsilon \left(\hat{f}\right). \end{array}$$

In the formula, Δ*R*=*x*_*p*_sin  *θ*_*m*,*k*_+*y*_*p*_Φ_*P*_, Φ_*B*_, represent the phase error caused by the translation between the transition assists and the phase error caused by the translation between the transition assist strings in turn in the carbon dioxide emission reduction analysis.

The article "Investigating the Impact of Transportation Infrastructure and Tourism on Carbon Dioxide Emissions in China" was retracted in 2023. Reasons: unreliable results or conclusions; concerns about the data; concerns about the peer review; concerns about the citations.

The realization of real-time, rational, and precise monitoring of carbon dioxide emissions can also provide a theoretical basis for the decision analysis of relevant environmental protection inspection departments, which is of great significance to the emergence of more transportation infrastructure projects. A detailed analysis of the transportation infrastructure is carried out to explore the problems and shortcomings of the carbon dioxide emission process so that the training and improvement plan can be formulated later. In the traditional CO_2_ emission evolution analysis process, CO_2_ emissions and real-time risk alerts are also effective data collection and analysis processes for CO_2_ emission devices. Collect indicator data and give feedback from the CO_2_ emission process. The obtained data are used to analyze the performance of carbon dioxide emission, analyze the operation state of carbon dioxide emission, and diagnose the cause of failure and can also be used to monitor the cause of failure. Carbon dioxide emissions and real-time risk alerts are an important manifestation of carbon dioxide emissions management and system integration, providing detailed data information for the operation and maintenance of carbon dioxide emissions [22, 23]. For transportation infrastructure, the development of tourism and carbon emissions has attracted more attention from researchers and scholars. Facts have proved that there are large gaps in carbon emissions changes under different environments and systems. Transportation carbon emission estimation is mainly through the use of life cycle assessment methods to estimate the carbon emissions generated by the constructed transportation infrastructure, and many researchers have developed carbon measurement software. The main theories and basic calculation ideas are relatively unified, but due to different divisions in different links, the coefficient library is not unified, the later detection is restricted insufficiently, and the existing carbon emission calculation methods of infrastructure equipment are disordered and have poor reference.

## 4. Analysis of Examples and Results

The continuous development of social economy promotes the continuous improvement of people's travel awareness. For the research on carbon dioxide emission reduction awareness of general tourists, carbon dioxide emission reduction awareness is the key internal driving force for tourists to implement environmental protection behaviors and proenvironmental behaviors. The disclosure of its influencing factors will undoubtedly play a positive role in improving the environmental protection behaviors of Chinese tourists. The environmental protection behaviors are classified and sorted, the influencing factors affecting tourists' environmental protection behaviors are constructed, and the relevant policies and measures of the existing Chinese tourists' environmental protection behaviors are sorted out and analyzed. Combined with the results of empirical analysis, targeted policy recommendations are put forward to promote the promotion of Chinese tourists' environmental protection concepts and behavior internalization. Because the driving force of tourism development is mainly labor-intensive industries, the impact of population size on carbon dioxide emissions is more serious [24]. However, with the continuous development of the regional tourism development level, the proportion of labor-intensive industries has gradually decreased, and the proportion of capital-intensive and high-tech related industries has gradually increased. The change of the influence coefficient of tourism consumption on carbon dioxide emissions follows the trend of first increase and then decrease. The influence coefficient of countries with a medium level of tourism development is the most significant, and countries with a low level of tourism development are less influential than countries with a high level of tourism development. Low-carbon resource technologies are generally better than other regions, and carbon dioxide emissions show a decreasing trend under the influence of the level of tourism development. It shows that in countries with backward tourism development, it is mainly necessary to use more resources and the environment in high-speed development as the price of development.

The article "Investigating the Impact of Transportation Infrastructure and Tourism on Carbon Dioxide Emissions in China" was retracted in 2023. Reasons: unreliable results or conclusions; concerns about the data; concerns about the peer review; concerns about the citations.

In this paper, we can use expression (17) to derive Ω in the assessment of CO_2_ emission limits using the growth rate of tourism to obtain the following expression:

(17) $$\begin{array}{c} \frac{d\left[\dot{P}/Y\right]}{d\Omega }=\delta^{-\varphi }{\left(1-\alpha \right)}^{\left(2\left(1-\alpha \right)\varphi /\alpha \right)}{\left(\delta L-\Omega \right)}^{\varphi -1}{\left(\rho +\Omega \right)}^{-\left(1-\alpha /\alpha \right)\left(\varphi -1\right)}\\ \times \;\left\{\left[\left(\frac{1-\alpha }{\alpha }-1\right)\varphi -1\right]\Omega^{2}+\left[\delta L\left(1-\frac{1-\alpha }{\alpha }\varphi \right)-\rho \left(1+\varphi \right)\right]\Omega +\delta \rho L\right\}. \end{array}$$

According to expression (24), if ((1 − *α*/*α*) − 1)*φ* − 1 < 0 is satisfied, then the relationship between the growth rate of the green economy and the carbon dioxide emission limit can be represented by an inverted *U* shape. *Q* is used to represent the horizontal axis and $d\left[\dot{P}/Y\right]/d\Omega$ to represent the vertical axis, then the corresponding intercept of expression (24) on the vertical axis is not less than zero. If ((1 − *α*/*α*) − 1)*φ* − 1 < 0 is satisfied, then the relationship between *δL*(1 − (1 − *α*)*φ*/*α*) − *ρ*(1 + *φ*) and 0 has a certain influence on the horizontal axis value corresponding to the extreme point of expression (24), according to three different situations shown in Figure 2. If *δL*(1 − (1 − *α*/*α*)*φ*) − *ρ*(1 + *φ*) < 0, 0 is satisfied, then it corresponds to Case 1 in Figure 2; if *δL*(1 − (1 − *α*/*α*)*φ*) − *ρ*(1 + *φ*) = 0 is satisfied, then it corresponds to Case 2; if *δL*(1 − (1 − *α*/*α*)*φ*) − *ρ*(1 + *φ*) > 0 is satisfied, then it corresponds to Case 3 in Figure 2. In the three cases in Figure 3, if the tourist growth rate Ω > 0 is satisfied, the intersection of expression (24) with the horizontal axis in the interval not less than 0 is set to Ω^*∗*^ in this paper. It can be concluded that if 0 < Ω < Ω^*∗*^$d\left(\dot{P}/Y\right)/d\Omega >0$, the growth rate of the green economy keeps rising, and the carbon dioxide emissions also increase; If Ω > Ω^*∗*^ is satisfied, $d\left[\dot{P}/Y\right]/d\Omega <0$, then the growth rate of the green economy will also rise, and carbon dioxide emissions will continue to decline. If Ω = Ω^*∗*^, $d\left[\dot{P}/Y\right]/d\Omega =0$, then the carbon dioxide emission will reach a maximum value at this time. According to the constructed model variables, ((1 − *α*/*α*) − 1)*φ* − 1 < 0 conforms to the standard of ecotourism economic development. In the expression (14) used, *α* represents the share of economic income in the total income. According to the green economy income share, it generally needs to be maintained between 60% and 70%, (1 − *α*)/*α* < 1 can be obtained, and the conditions of ((1 − *α*/*α*) − 1)*φ* − 1 < 0 need to be met.

The article "Investigating the Impact of Transportation Infrastructure and Tourism on Carbon Dioxide Emissions in China" was retracted in 2023. Reasons: unreliable results or conclusions; concerns about the data; concerns about the peer review; concerns about the citations.

According to the above detailed analysis, this paper uses quantitative analysis to obtain the impact of ecotourism and transportation infrastructure on Chinese carbon dioxide emissions. According to the constructed expression, the explanatory variables serve as the effect of limiting carbon dioxide emissions, and the core explanatory variables mainly include the level of ecotourism and transportation infrastructure. Combining the model, we can effectively calculate the basic impact of ecotourism on carbon dioxide emissions. Therefore, this paper can analyze the factors affecting carbon dioxide emissions in detail. Due to the large differences in regional economic growth, according to the regional economic development level and carbon dioxide emissions of each country, based on the actual situation, the reasonable and scientific carbon emission reduction policy standards are formulated, which has become the first choice for the development of low-carbon economy in China. When countries formulate low-carbon emission reduction policies, they need to comprehensively consider their own economic development, basic social conditions, energy availability, and green-related policies, actively encourage Chinese exploration of carbon dioxide emissions and renewable energy quotas suitable for their own regions, and guide the whole society to save energy and improve energy efficiency to reduce environmental pollution.

## 5. Conclusions

In the future, the scale of transportation infrastructure construction is expected to continue to expand, and the carbon emissions generated during its construction need further attention. This paper focuses on the impact of carbon dioxide emissions on tourism development areas. The speed of tourism development is directly related to carbon emissions. The development of low-carbon life is mandatory, and real improvements are made from the way of carbon reduction. This improvement determines the quality of the living environment and is a powerful manifestation of a sense of social responsibility. A comprehensive model of ecotourism, transportation infrastructure, and carbon dioxide emissions is constructed. Compared with traditional policies and regulations, in the proportion of large-scale investment in ecotourism, economic competition, and transportation infrastructure, carbon dioxide emissions are greatly reduced. The long-term development of the Chinese economy has a positive driving effect, which can not only effectively accelerate economic growth but also optimize the economic structure of ecotourism. At present, Chinese general environment has entered a new course, and the development of tourism in each region is different, which plays a decisive role in local carbon emissions. Improving the status quo requires lower carbon, greener, and less energy consumption to generate maximum tourism benefits.

## Figures and Tables

**Figure 1:** Main links of carbon emissions from transportation infrastructure.

**Figure 2:** CO_2_ emission control strategy formulation process.

**Figure 3:** Visual analysis of the impact of the tourism growth rate on carbon dioxide emissions.

**Table 1:** Carbon emission coefficient of conventional resources.

Types of resources	Carbon emission factor (kg·(c)/kg)
Liquified petroleum gas	0.5034
Diesel oil	0.5933
Gasoline	0.5535
Fuel oil	0.6144
Oil	0.54/0.577
Electricity^*∗*^	0.26/0.276
Coal	0.68/0.755

^*∗*^The unit is kg (c)·kW·h.

The article "Investigating the Impact of Transportation Infrastructure and Tourism on Carbon Dioxide Emissions in China" was retracted in 2023. Reasons: unreliable results or conclusions; concerns about the data; concerns about the peer review; concerns about the citations.

**Table 2:** Carbon emission coefficients of main building materials.

Type of material	Steels	Ready-mixed concrete	Cement	Concrete brick block	Wooden product
Carbon emission coefficient (*t*/*t*)	2.1	0.25 *t*/m^3^	0.81	0.13	0.21

## Data Availability

The data used to support the findings of this study are available from the corresponding author upon request.
